The article "Gender Discrepancy in Patients with Traumatic Brain Injury: A Retrospective Study from a Level 1 Trauma Center" was published in 2022. Journal: Biomed Res Int.

# Gender Discrepancy in Patients with Traumatic Brain Injury: A Retrospective Study from a Level 1 Trauma Center

**DOI:** 10.1155/2022/3147340

**Published:** 2022-08-18

**Authors:** Ayman El-Menyar, Ahammed Mekkodathil, Vishwajit Verma, Bianca M. Wahlen, Ruben Peralta, Ibrahim Taha, Suhail Hakim, Hassan Al-Thani

**Affiliations:** ^1^Clinical Research, Trauma & Vascular Surgery, Hamad General Hospital, Doha, Qatar; ^2^Clinical Medicine, Weill Cornell Medical College, Doha, Qatar; ^3^Trauma Surgery Section, Hamad General Hospital (HGH), Doha, Qatar; ^4^Department of Anesthesia, Hamad General Hospital (HGH), Doha, Qatar; ^5^Department of Surgery, Universidad Nacional Pedro Henriquez Urena, Santo Domingo, Dominican Republic

## Abstract

**Objectives:**

The objective of this study is to explore the gender discrepancy in patients with traumatic brain injury (TBI).

**Methods:**

A retrospective analysis of Qatar Trauma Registry (QTR) was conducted among patients (age ≥14y) who were hospitalized with TBI. Data were collected and analyzed based on the gender and age.

**Results:**

Over 5 years (2014-2019), 9, 309 trauma patients (90% males and 10% females) were admitted to the trauma center. Of these, 1, 620 (17.4%) patients were hospitalized with TBI (94% males and 6% females). Motor vehicle crash was the main mechanism of injury (MOI) in females, and fall from height was predominant among males. Subdural hematoma (SDH) was the more frequent type of TBI in both genders, but it was more prevalent in male patients ≥55 years. Injury severity score, Glasgow coma scale, and head abbreviated injury score were comparable between males and females. The length of stay in the ICU and hospital and mortality were similar in both genders. However, mortality was higher among males ≥55 years when compared to 14-54 years within the same gender (21% vs. 12%, *p* = 0.002). The crude and adjusted odds ratio did not show that gender is a significant predictor of mortality among TBI patients.

**Conclusions:**

Although the incidence and MOI of TBI show significant differences between male and female patients, the severity and outcomes are comparable.

## 1. Introduction

Traumatic brain injury (TBI) could result from a forceful blow or jolt to the head, body, or a penetrating trauma to the brain tissue which leads to disruption of the normal functions of the brain [1]. It remains a major public health problem worldwide, causing substantial losses to individuals, families, and communities [2]. TBI patients may die or lead a life with permanent disabilities requiring long-term care and therefore incur social and economic burden [2, 3]. Falls and motor vehicle crashes (MVCs) are the two leading causes of TBI-related hospitalizations, and intentional self-harm is the main cause of TBI-related deaths [4]. In the USA, TBI-related emergency department (ED) visits, hospitalizations, and deaths occurred in 2014 was estimated as 2.87 million, of which TBI mortality was 56,800 (2%) [4]. In the Middle East region, the median TBI incidence rate was estimated as 45 per 100,000 population, and the TBI-related mortality in ED and intensive care unit (ICU) was estimated as 10% and 25%, respectively [5]. A recent systematic review from the Middle East and North Africa (MENA) region reported a TBI mortality rate of 13% [6].

The article "Gender Discrepancy in Patients with Traumatic Brain Injury: A Retrospective Study from a Level 1 Trauma Center" was published in 2022. Journal: Biomed Res Int.

Although both genders are affected, evidence suggests that gender can influence cognitive impairment, short- and long-term outcomes, and mortality associated with TBI [5]. Previous reports have shown male predominance [7, 8] in TBI due to increased probability of injuries; however, females were shown to have worse outcomes when compared to males [9]. In contrast, a retrospective review of the National Trauma Data Bank (NTDB) in the USA revealed that female gender was independently associated with reduced mortality and decreased complications following TBI [10]. The present study aims to explore the effect of gender on the incidence, presentation, management, and outcomes of TBI based on a subanalysis of the trauma registry data from a level 1 trauma center from a Middle Eastern country.

## 2. Methods

A retrospective analysis of the Qatar Trauma Registry (QTR) was conducted among patients who were admitted to the Hamad Trauma Center (HTC) following TBI. The QTR is compliant with both the National Trauma Data Bank [NTDB] and Trauma Quality Improvement Program [TQIP] of the American College of Surgeons-Committee on Trauma and has regular internal and external validations [11]. Injuries were defined according to the International Classification of Diseases (ICD-10 codes). The abbreviated injury severity score (AIS), injury severity score (ISS), and Glasgow coma score (GCS) were described previously [12]. TBI was defined as head abbreviated injury severity scale (AIS) ≥1. The HTC is the only level 1 trauma care facility in the country which treats patients with moderate to severe injuries. The study duration was between January 2014 and February 2019. All patients with age ≥14 years admitted due to TBI were included in the study. Patients with age <14 years, dead on arrival, and dead within 24 hours or transferred from or to other facility were excluded. Patients with missing relevant data were also excluded. The collected data included age; gender; types of TBI; mechanism of injury; associated injuries; AIS; ISS; GCS; intubation; ventilator days; ventilator associated pneumonia (VAP); hospital length of stay (LOS); and in-hospital mortality. Types of TBI data include subdural hematoma (SDH); epidural hematoma (EDH); subarachnoid hemorrhage (SAH); contusion; diffuse axonal injury (DAI); and edema. Data were compared between the two gender groups and by age groups within the gender. The age groups in females capture the pre- and postmenopausal periods, i.e., 14-54 years and ≥55 years, respectively.

The article "Gender Discrepancy in Patients with Traumatic Brain Injury: A Retrospective Study from a Level 1 Trauma Center" was published in 2022. Journal: Biomed Res Int.

Statistical analysis: Data were expressed as numbers, percentages, mean ± standard deviation, or medians with interquartile range whenever appropriate. Chi-square test was performed for the analysis of differences in categorical variables between gender groups, and Fisher exact test was used when observed cell values *n* < 5. The continuous variables between different groups were compared using Student's *t* test. Crude and adjusted odds ratio (OR) for prediction of mortality were performed and data expressed as OR and 95% confidence interval (CI). Two-tailed *p* values <0.05 were considered as significant. Data analysis was carried out using the Statistical Package for Social Sciences version 26 (SPSS Inc. Chicago, IL, USA). The population data was available from the Planning and Statistics Authority, Qatar website, used to calculate TBI incidence rates over the years [13].

## 3. Results

During the study duration between 2014 and 2019 (5 years), a total of 9,309 patients (8370 (90%) males and 939 (10%) females) were admitted to the HTC. Of these, 1,620 (17.4%) patients were hospitalized due to TBI. The proportion of males and females with TBI admissions was 18.3% (1529/8370) and 9.7% (91/939), respectively (*p* = 0.001). Of the TBI patients, 94% were males and 6% females. Further analysis based on age groups within the gender revealed that males under the age of 55 years were more predominant TBI victims.  Table 1 shows the characteristics, management, and outcomes of TBI patients admitted at HTC by gender.

Motor vehicle crash (MVCs) was the main mechanism of injury in females when compared to males (43% vs.29%, *p* = 0.04). Furthermore, females under the age of 55 years were the majority of the MVC victims (50% of females). On the other hand, fall from height (FFHs) was the major contributor among injured males compared to females (35% vs. 26%, *p* = 0.04). Males and females older than 54 years of age were proportionately higher among fall victims (53% and 62%, respectively, in each group). Chest, abdominal, and musculoskeletal injuries among both genders were comparable. Musculoskeletal injuries were more common in premenopausal females (56%) and males under the age of 55 years (48%). Comorbidities (diabetes and hypertension) represented 11.8% of the cohort and were more prevalent among males than females.

The article "Gender Discrepancy in Patients with Traumatic Brain Injury: A Retrospective Study from a Level 1 Trauma Center" was published in 2022. Journal: Biomed Res Int.

Midline shift on the admission CT scan was present in 1 out of 5 patients with traumatic brain injury without any significant difference between the genders. SDH was the most encountered intracranial lesion, though there was no statistically significant difference in the frequency of intracranial lesions between genders. However, there was a significant difference in types of TBIs by age groups within the males. SDH was more prevalent in male patients older than 54 years. TBI types were comparable within the female age groups. Injury scores such as GCS, AIS, and ISS were similar among both genders. Within the males, GCS at ED among 14-54 years of age had significantly lower GCS when compared to males ≥55 years of age. The rate of intubation was similar in both genders; however, it was more frequent in the premenopausal females.  Table 2 shows patients characteristics, management, and outcomes of TBI by gender and age.

Outcomes including duration of being on mechanical ventilator, ICU, and hospital LOS were similar in both genders. In addition, there was no significant difference in the in-hospital mortality by gender. However, mortality was higher among males older than 54 years of age when compared to 14-54 years within the male group (21% vs. 12%, *p* = 0.002).

### 3.1. Predictors of Mortality

The crude (OR 1.06; 95% CI 0.57-1.99, *p* = 0.85) and adjusted odds ratio (OR 0.98; 95% CI 0.47-2.06, *p* = 0.96) did not show significant association between gender and mortality among TBI patients. The multivariate regression analysis showed that age, ISS, and head AIS were the predictors of mortality after adjusting for gender and comorbidity (Table 3).

## 4. Discussion

The present study estimated that one out of six trauma admissions in Qatar had moderate to severe TBI. TBI-related hospitalizations were significantly higher among males when compared to females. Although the mechanism of injuries differed by gender, the type of TBI lesion and other associated injuries and injury severities were comparable. Moreover, there were no significant differences in outcomes such as hospital LOS and in-hospital mortality by genders. Further analysis based on age groups within the genders revealed that females <55 years of age were more likely to be involved in MVCs, while females ≥55 years were more frequently involved in fall-related injuries. Within the males, SDH was more frequent among males ≥55 years. This higher rate of acute traumatic SDH among males than females was also reported in many previous studies from different countries. For instance, the proportions of affected males were 52% (Portugal), 53% (Italy and Spain), 64% (Japan), 65% (the USA), and 74% (Brazil) [14–18]. However, there is no reported explanation in the literature for such gender discrepancy. In traumatic SDH, gender was not influencing the hospital survival [15–18]; however, male gender was associated with a poor functional outcome in one study [14]. Although in-hospital mortality was comparable by gender, males ≥55 years had a higher mortality rate when compared to young age males in our study. Crude and adjusted OR did not show that gender is a predictor of mortality among TBI patients. On the contrary, a recent study in 2021 from Japan showed that the adjusted OR of TBI mortality for males in comparison to females was 1.32 (95% CI 1.22-1.42) [19]. Moreover, this gender difference impact was evident in the age group of 10-19 years and those who aged 65 and above. A previous study from the USA in 2000 showed that crude OR showed that increasing age, but not the gender was a predictor of mortality; however, after adjusting for age, GCS, ISS, and type of trauma (penetrating vs blunt), female gender was a predictor of mortality with OR 1.75 [20].

The article "Gender Discrepancy in Patients with Traumatic Brain Injury: A Retrospective Study from a Level 1 Trauma Center" was published in 2022. Journal: Biomed Res Int.

Male predominance in TBI incidence was shown in previous studies [5–7] which is in line with increased probability of males to getting injured due to differences in sociological attributes and growing environment [21]. Our study sample size (*n* = 1,620) was comparable to a previous retrospective study by Munivenkatappa et al. on gender-related TBI outcomes which included 1627 patients [22]. However, the proportion of females in their study was higher compared to our study (20% vs. 6%) [22]. The male to female ratio in TBI cases in our study was 16.8 : 1 (i.e., one female TBI case for every 17 male TBI cases). The population estimates from Qatar shows that the proportion of the male population is nearly 3 times higher than females and is over 3 times for age>14 years [13]. In addition to the fact that males are more prone to injuries, Qatar's unique population and workforce structure with vast majority of migrant workers, mainly young and middle-aged males, involved in high-risk jobs especially in the construction sector, making them more susceptible to head injuries than females [23, 24]. Blunt trauma in Qatar comprises more than two thirds of trauma-related hospitalizations and 90% of patients are young males [11, 25, 26].

Although several studies reported worse clinical outcomes in women when compared to men, gender-related TBI outcomes remain controversial [7–10]. After TBI in 439 patients, Leitgeb et al. concluded that gender had no significant effect on the hospital outcome, although the mortality was 7% higher in females, and this difference was mainly related to the age and severity of CT scan findings [8]. Munivenkatappa et al. found that female TBI patients presented with worse GCS and the mortality rate were significantly higher compared to males (3.4% vs. 1.6%) in Indian population [22]. A Singapore-based study of severe TBI cases also found significantly higher mortality in females when compared to males [27]. Female patients in this study were older than males (54 vs. 43 years, *p* = 0.001), though this difference was not significant when adjusted for GCS, the presence of multiple injuries and postresuscitation pupillary abnormalities [27]. These findings are in contrast with our results which demonstrate comparable in-hospital mortality rate by gender. In our study, males and females differed only in terms of age and mechanism of injuries. The Singapore study also demonstrated that females aged 60 and below were more likely to have a poorer outcome when crude and adjusted odd ratios were considered [27]. In our study, further analysis among TBI females by age categories revealed comparable outcomes. However, mortality rate was significantly higher among older males when compared to the young and middle-aged males. In contrast to the studies from the Asian population, a USA-based study on moderate to severe TBI cases reported that females had a significantly lower risk in mortality and in developing complications than the male population [10]. The authors concluded poor outcomes in premenopausal women when compared to perimenopausal and postmenopausal women [10]. Phelan et al. found that female gender was associated with improved survival rates in the postpubescent age group (14.5–20 years), while Davis et al. reported improved outcomes in postmenopausal patients [28, 29]. On the other hand, Coimbra et al. found no significant differences in TBI outcomes under the age of 50 years [30]. Many confounding factors like severity of TBI, age, and physical condition of the patients could play a role in the TBI outcomes [31–34]. Improved survival among the premenopausal women reported in some studies could be related to the effect of female sex steroids levels after TBI [21]. Sex hormones might reduce the intracerebral pressure and improve the cerebral perfusion pressure [19, 35]. Although a meta-analysis revealed poorer outcome in females sustaining severe TBI than males, few studies reported better outcome after administration of progesterone, properly due to its effect as it reduces the cerebral edema and promotes a neuroprotection [9, 14, 35–37]. Progesterone has a membrane stabilizing effect and may suppress the neuronal hyperexcitability after trauma [37]. Furthermore, the estrogen hormone is a potent antioxidant, preserves autoregulatory functions, reduces neuronal excitotoxicity, activates the mitogen-activated protein kinase (MAPKs), and upregulates the antiapoptosis (that prevents cell loss) in females after injury [37]. A recent larger study from Japan on patients sustaining isolated TBI found that, among younger and older populations, male gender was associated with higher mortality compared to females [19]. However, differences in mortality after TBI by gender remain inconclusive in the literature. A subanalysis of CRASH-3 study on TBI patients (but with small sample size) showed that females (*n* = 21) were receiving less tranexamic acid than males (*n* = 91) and the relative risk of death was only significantly better in males [38]. Therefore, we cannot advocate specific early treatment (i.e., administration of tranexamic acid or hormonal therapy) based only on gender discrepancy until larger multicenter studies addressing the causation and not only the association.

The article "Gender Discrepancy in Patients with Traumatic Brain Injury: A Retrospective Study from a Level 1 Trauma Center" was published in 2022. Journal: Biomed Res Int.

### 4.1. Limitations

This study has several limitations due to the retrospective study design , ad hoc analysis and single trauma center experience that may not be applicable or generalizible to other settings. However, the study is a representative of the country trauma patients as data are retrieved from the HTC; the only level 1 tertiary trauma center admits and treats around 95% of injuries in Qatar. The HTC has an internal and external regular validation and linked to the National Trauma Data Bank (NTDB) and compliant with the standards of the American College of Surgeons Trauma Quality Improvement Program (ACS-TQIP) in the USA. Of note, based on the Qatar population, the male to female ratio is 3 : 1, whereas the trauma-related hospitalization ratio is 9 : 1 [5, 11]. Disproportionate number of male and female patients is a limitation. The small number of females might be misrepresentative of this gender; however, this limitation has been observed in the majority of prior studies. The outcome after TBI might be influenced by patient's comorbidity such as diabetes mellitus, hypertension, dyslipidemia, smoking, chronic obstructive pulmonary disease, and heart disease; however, our data could be unique in terms of patient age in comparison to prior studies from other countries [14–18] as the mean age in our cohort is 34 ± 14 which precludes the presence of high proportion of comorbidities. However, diabetes mellitus and hypertension were found in 11.8%, and multivariate analysis showed that they did not have a significant predictor role for mortality. Other comorbidities were not captured in this analysis.

The article "Gender Discrepancy in Patients with Traumatic Brain Injury: A Retrospective Study from a Level 1 Trauma Center" was published in 2022. Journal: Biomed Res Int.

## 5. Conclusions

Although, the incidence and MOI of TBI show significant differences between male and female patients, the severity and outcomes seem comparable. Further multicenter studies are required to support these findings and to consider the other confounding factors.

## Figures and Tables

**Table 1:** Characteristics, management and outcomes of traumatic brain injury (TBI) patients admitted at Hamad Trauma Center stratified by gender.

	Overall (*N* = 1620)	Male (*n* = 1,529, 94.4%)	Female (*n* = 91, 5.6%)	*p* value
Age in years ±SD	34.4 ± 13.9	34.1 ± 13.5	39.9 ± 18.5	0.004
*Mechanism of injury (%)*				
Motor vehicle crashes	486 (30.0)	447 (29.2)	39 (42.9)	0.04 for all
Fall from height	551 (34.0)	527 (34.5)	24 (26.4)	
Pedestrian	268 (16.5)	257 (16.8)	11 (12.1)	
Other mechanisms	315 (19.4)	298 (19.5)	17 (18.7)	
Comorbidities^∗^ (%)	192 (11.8%)	174 (90.6%)	18 (9.4%)	0.048
*Injuries (%)*				
Chest	594 (36.7)	559 (36.6)	35 (38.5)	0.71
Abdominal	203 (12.5)	187 (12.2)	16 (17.6)	0.13
Musculoskeletal	768 (47.4)	725 (47.4)	43 (47.3)	0.98
*Type of TBI (%)*				
(i) SDH	434 (26.8)	406 (26.6)	28 (30.8)	0.09
(ii) EDH	366 (22.6)	354 (23.2)	12 (13.2)	
(iii) Contusion	294 (18.1)	276 (18.1)	18 (19.8)	
(iv) SAH	131 (8.1)	119 (7.8)	12 (13.2)	
(v) DAI	118 (7.3)	110 (7.2)	8 (8.8)	
(vi) Edema	103 (6.4)	101 (6.6)	2 (2.2)	
(vii) Others	174 (10.7)	163 (10.7)	11 (12.1)	
(viii) Midline shift	360 (22.2)	342 (22.4)	18 (19.8)	0.56
*Injury characteristics*				
GCS at ED	14 IQR (3-15)	14 IQR (3-15)	14 IQR (3-15)	0.74
Median AIS head	3 IQR (3-5)	3 IQR (3-5)	3 IQR (3-4)	0.44
ISS	22 IQR (14-29)	22 IQR (14-29)	19 IQR (13-27)	0.55
Intubation (%)	772 (47.7)	735 (48.1)	37 (40.7)	0.17
*Ventilator days*				
(i) >7 days	396 (24.4)	379 (24.8)	17 (18.7)	0.32
(ii) ≤7 days	376 (23.2)	356 (23.3)	20 (22.0)	
(iii) Not intubated	848 (52.3)	794 (51.9)	54 (59.3)	
Ventilator-associated pneumonia (%)	169 (10.4)	156 (10.2)	13 (14.3)	0.22
*Outcomes*				
LOS	10 IQR (5-22)	10 IQR (5-22)	10 IQR (4-25)	0.73
LOS>30 days (%)	261 (16.1)	243 (15.9)	18 (19.8)	0.33
Mortality (%)	203 (12.5)	191 (12.5)	12 (13.2)	0.85

TBI: traumatic brain injury; SDH: subdural hematoma; EDH: epidural hematoma; SAH: subarachnoid hemorrhage; DAI: diffuse axonal injury; GCS: Glasgow coma score; ED: emergency department; AIS: abbreviated injury score; ISS: injury severity score; LOS: length of stay, comorbidities^∗^ = diabetes or hypertension or both.

**Table 2:** Characteristics, management and outcomes of TBI patients by gender and age (*N* = 1620).

	Males (*n* = 1,529)			Females (*n* = 91)		
	Age 14-54 yrs (*n* = 1, 401, 91.6%)	Age ≥55 yrs (*n* = 128, 8.4%)	*p* value	Age 14-54 yrs (*n* = 70, 76.9%)	Age ≥55 yrs (*n* = 20, 23.1%)	*p* value
*Mechanism of injury*						
Motor vehicle crashes	418 (29.8)	29 (22.7)	0.001	35 (50.0)	4 (19.0)	0.001 for all
Fall from height	459 (32.8)	68 (53.1)		11 (15.7)	13 (61.9)	
Pedestrian	235 (16.8)	22 (17.2)		9 (12.9)	2 (9.5)	
Other mechanisms	289 (20.6)	9 (7.0)		15 (21.4)	2 (9.5)	
*Injuries*						
Chest	510 (36.4)	49 (38.3)	0.67	30 (42.9)	5 (23.8)	0.12
Abdominal	173 (12.3)	14 (10.9)	0.64	15 (21.4)	1 (4.8)	0.08
Musculoskeletal	676 (48.3)	49 (38.3)	0.03	39 (55.7)	4 (19.0)	0.003
*Type of TBI*						
(i) SDH	346 (24.7)	60 (46.9)	0.001	17 (24.3)	11 (52.4)	0.17 for all
(ii) EDH	343 (24.5)	11 (8.6)		10 (14.3)	2 (9.5)	
(iii) Contusion	259 (18.5)	17 (13.3)		17 (24.3)	1 (4.8)	
(iv) SAH	102 (7.3)	17 (13.3)		9 (12.9)	3 (14.3)	
(v) DAI	99 (7.1)	11 (8.6)		7 (10.0)	1 (4.8)	
(vi) Edema	98 (7.0)	3 (2.3)		1 (1.4)	1 (4.8)	
(vii) Others	154 (11.0)	9 (7.0)		9 (12.9)	2 (9.5)	
(viii) Midline shift	307 (21.9)	35 (27.3)	0.15	12 (17.1)	6 (28.6)	0.25
*Injury characteristics*						
GCS at ED	13 IQR (3-15)	15 IQR (10-15)	0.001	13 IQR (3-15)	15 IQR (13-15)	0.60
Median AIS head	3 IQR (3-5)	4 IQR (3-5)	0.45	3 IQR (3-5)	3 IQR (3-4)	0.99
Injury severity score	22 IQR (14-29)	19 IQR (12-29)	0.39	22 IQR (14-29)	17 IQR (10-20)	0.05
Intubation	684 (48.8)	51 (39.8)	0.05	33 (47.1)	4 (19.0)	0.02
*Ventilator days*						
(i) >7 days	353(25.2)	26 (20.3)	0.15	15 (21.4)	2 (9.5)	0.07 for all
(ii) ≤7 days	331 (23.6)	25 (19.5)		18 (25.7)	2 (9.5)	
(iii) Not intubated	717 (51.2)	77 (60.2)		37 (52.9)	17 (81.0)	
Ventilator-associated pneumonia	145 (10.3)	11 (8.6)	0.53	12 (17.1)	1 (4.8)	0.16
*Outcomes*						
LOS	10 IQR (5-22)	9 IQR (4-26)	0.45	11 IQR (5-26)	6 IQR (4-11)	0.35
LOS>30 days	217 (15.5)	26 (20.3)	0.15	15 (21.4)	3 (14.3)	0.47
Mortality	164 (11.7)	27 (21.1)	0.002	8 (11.4)	4 (19.0)	0.37

SDH: subdural hematoma; EDH: epidural hematoma; SAH: subarachnoid hemorrhage; DAI: diffuse axonal injury; GCS: Glasgow coma score; ED: emergency department; AIS: abbreviated injury score; ISS: injury severity score; LOS: length of stay.

The article "Gender Discrepancy in Patients with Traumatic Brain Injury: A Retrospective Study from a Level 1 Trauma Center" was published in 2022. Journal: Biomed Res Int.

**Table 3:** multivariable logistic regression analysis for predictors of mortality among TBI patients.

Predictor	*p* value	Odds ratio	95% confidence intervals
Gender	0.640	1.192	0.571-2.490
Age	0.001	1.023	1.010-1.037
Injury severity score	0.001	1.080	1.052-1.106
Head abbreviated injury severity (AIS)	0.001	1.810	1.323-2.477
Comorbidities (DM and hypertension)	0.550	0.783	0.351-1.746

## Data Availability

All data were presented in the manuscript and tables.

## Abbreviations

ISS: Injury severity score
AIS: Abbreviated injury scale
GCS: Glasgow coma scale
TBI: Traumatic brain injury.
